The article "The Design of the Lightweight Smart Home System and Interaction Experience of Products for Middle-Aged and Elderly Users in Smart Cities" was published in 2022. Journal: Comput Intell Neurosci.

# The Design of the Lightweight Smart Home System and Interaction Experience of Products for Middle-Aged and Elderly Users in Smart Cities

**DOI:** 10.1155/2022/1279351

**Published:** 2022-06-15

**Authors:** Qingnan Ji

**Affiliations:** Department of Art and Design, Shaanxi Fashion Engineering University, Xi'an City 710000, China

## Abstract

The research aims to improve the comfort and safety of the smart home by adding a motion recognition algorithm to the smart home system. First, the research status of motion recognition is introduced. Second, based on the requirements of the smart home system, a smart home system is designed for middle-aged and elderly users. The software system in this system includes intelligent control subsystems, intelligent monitoring subsystems, and intelligent protection subsystems. Finally, to increase the security of the smart home, the intelligent monitoring subsystem is improved, and an intelligent security subsystem is proposed based on a small-scale motion detection algorithm. The system uses three three-dimensional (3D) convolutional neural networks (CNNs) to extract three image features, so that the data information in the video can be fully extracted. The performance of the proposed intelligent security subsystem based on a small-scale motion detection algorithm is compared and analyzed. The research results show that the accuracy of the system on the University of Central Florida (UCF101) dataset is 94.64%, and the accuracy on the HMDB51 dataset is 90.11%, which is similar to other advanced algorithms. Observing whether there are dangers such as falling inside and outside the family through motion recognition technology has very important application significance for protecting people's personal safety, life, and health.

## 1. Introduction 

With the continuous upgrading and transformation of information technology, the Internet of Things (IoT) has developed rapidly. Lv et al. [1] mentioned that the emergence of “smart cities” has brought convenience to people's lives. The smart city refers to the use of current advanced information technology and related innovative concepts to integrate various urban operation systems and service channels to improve the living standards of residents and the efficiency of social resource utilization [2–4]. It is said that developed countries such as the United States, Japan, and other developed countries have added household robots in their strategic plans for robot development. The housekeeping services provided by such robots will enter people's daily lives, which will lead to contact with robots becoming a part of human daily life. Research on human–computer interaction (HCI) will become a hot spot in the future [5]. Therefore, how to improve the existing methods of HCI so that machines can understand human behavior more accurately and intelligently has become a major focus of artificial intelligence (AI) research.

The article "The Design of the Lightweight Smart Home System and Interaction Experience of Products for Middle-Aged and Elderly Users in Smart Cities" was published in 2022. Journal: Comput Intell Neurosci.

At present, aging has become a global problem. Now China has entered the stage of aging of the population. Respecting and caring for the elderly has always been a fine tradition in China, and people will pay more attention to the life of the elderly. With the update of technology and the activeness of the smart home, the research on smart homes related to middle-aged and elderly users has attracted the attention of scholars, such as the auxiliary interactive building project in the United Kingdom in 1996, the consciousness home project in the United States in 1999, and the Tiger Palace project in France in 2003, the crocodile technology smart home project in the United States in 2004, and the robotic technology home environment project in Italy in 2007, these smart home projects are designed to improve the ability of the elderly to live alone and the safety of living alone [6, 7]. At present, smart homes are more intelligent and automated after combining cloud remote connection technology and wireless communication technology [8]. With the rapid development of intelligent monitoring technology, image recognition technology has gradually penetrated into the field of smart homes. In the future, more than half of home security monitoring products will add image recognition algorithms to improve the safety performance of products [9, 10]. In addition, security-monitoring products based on image recognition technology will become mainstream in future smart home systems. Such a product can accurately judge the user's identity and the shape of the human body at the same time, which will greatly improve the monitoring efficiency of the product and the user's interactive experience. With the rapid development of computer hardware technology, the performance of computers has been greatly improved, making deep learning (DL) technology widely used. Since the neural network (NN) model can automatically learn the feature information in the image, the workload of manual labeling is reduced and the NN model has better performance. In recent years, the research in the fields of image processing, face recognition, and action recognition has been occupied by algorithms based on NN, and deep features have gradually replaced manual features in various fields. Behavioral features learned based on deep convolutional neural networks (CNN) can automatically learn feature representations from big data, which can contain thousands of parameters. With more and more labeled behavior videos, it gradually surpasses manual features and becomes the mainstream behavior feature extraction method.

The article "The Design of the Lightweight Smart Home System and Interaction Experience of Products for Middle-Aged and Elderly Users in Smart Cities" was published in 2022. Journal: Comput Intell Neurosci.

The monitoring and HCI functions of image recognition in the smart home are deeply explored. The purpose of the research is to improve the comfort and safety of smart homes by adding motion recognition algorithms to smart home systems. A smart home system for middle-aged and elderly users is designed. The software system in this system includes three parts: intelligent control subsystem, intelligent monitoring subsystem, and intelligent protection subsystem. To increase the security of the smart home, the intelligent monitoring subsystem is improved, and an intelligent security subsystem based on a small-scale motion detection algorithm is proposed. The proposed intelligent security subsystem based on a small-scale motion detection algorithm can maximize the temporal and spatial features in the video, improve the performance of the algorithm, and realize the intelligent security function based on human motion. The research on motion recognition technology for intelligent monitoring has very vital application significance for protecting people's personal safety, life, and health.

## 2. Research Status of Action Recognition

The key steps of action recognition are basically similar to the key steps of image processing, both of which are the extraction of the feature first, followed by the classification of the feature. The extraction of action features is very significant for action recognition, and whether the action features in the video can be fully extracted directly affects the final effect of the recognition. Human action recognition involves human activity monitoring tasks in diverse fields such as medical care, education, entertainment, visual surveillance, video retrieval, and abnormal activity recognition [11, 12]. Therefore, in the course of more than 30 years of action recognition research, scholars have focused on how to fully extract action features from video recordings for better action classification. In the past, action features can be roughly divided into two categories: manual features and deep features. Now with the development of hardware technology, people can obtain more types of action features through specific equipment to identify human actions. Manual features can be divided into two categories: local features and global features. As DL methods have made major breakthroughs in the fields of image classification and target detection, many scholars have turned their attention to the research topic of obtaining more recognizable human behavior feature descriptors based on DL methods. Pareek and Thakkar [13] discussed various machine learning (ML) and DL techniques for human action recognition from 2011 to 2019, the characteristics of public datasets for human action recognition, and also introduced various action recognition techniques and an overview of applications of human action recognition. Namely, content-based video summarization, HCI, education, healthcare, video surveillance, abnormal activity detection, sports, and entertainment. Zhang et al. [14] proposed a cognitive computing system model based on Deep Belief Network (DBN) and applied it to the control system of collaborative robots.

The article "The Design of the Lightweight Smart Home System and Interaction Experience of Products for Middle-Aged and Elderly Users in Smart Cities" was published in 2022. Journal: Comput Intell Neurosci.

Vision-based human action recognition has been a research hotspot in the last decade because of its popular applications such as visual surveillance and robotics. To correctly recognize actions, various local and global points need to be referred to as features, which change with human motion [15]. Due to the subtle variation of several human actions, the features of these actions are mixed, which degrades the recognition performance. Therefore, Khan et al. [16] designed a new 26-layer CNN structure for accurate recognition of complex actions, extracted features from global average pooling layers and fully connected layers. They fused through the proposed high-entropy-based method and also proposed a feature selection method-Poisson distribution and univariate measure. Compared with the existing techniques, the structure has better performance in terms of accuracy and test time. Human action recognition, and video summarization are a challenging task for multiple computer vision applications including video surveillance, criminal investigation, and sports applications. For long videos, it is difficult to search for a specific action and/or person in the video. Human action recognition methods deal with videos that contain only one person, and the method can identify his actions. Elharrouss et al. [17] put forward an efficient multiperson action detection, recognition, and summarization method. Multiaction detection extracts human silhouettes and then uses motion detection and tracking methods to generate specific sequences for each human. Using the similarity between each pair of frames, each extracted sequence is divided into shots representing homogeneous actions in the sequence. Actions are identified using the proposed CNN model, performing an action summary for each detected person. The experimental results indicate that the method can detect and recognize multiple actions well.

Compared with manual features, behavioral features based on deep learning are automatically learned by machines. On the one hand, the design burden of artificial features is reduced. On the other hand, a properly designed deep model not only has powerful learning ability, but its expressive ability also is more efficient than traditional models. The depth model can extract information features layer by layer from pixel-level raw data, and finally obtain abstract language concepts and analyze human behavior information. Based on the above analysis, due to the development of DL technology, CNN can be used to solve some practical problems, such as image classification, video analysis, whose video data features are learned in an end-to-end manner. Some past studies trained 2D-CNN to recognize human actions, but still images contain very limited information, and 2D-CNN cannot fully extract action information in videos. To improve the recognition degree of the original optical flow image and mine the more diverse human action information in the video, a new action recognition system is proposed. The system consists of three 3D-CNN models, which can fully extract action information in videos.

The article "The Design of the Lightweight Smart Home System and Interaction Experience of Products for Middle-Aged and Elderly Users in Smart Cities" was published in 2022. Journal: Comput Intell Neurosci.

## 3. Design of Lightweight Smart Home System for Middle-Aged and Elderly Users

### 3.1. Demand Analysis of Smart Home System

Smart home system is an environmental system composed of intelligent control module products and home furnishing, which can provide a convenient, comfortable, and safe home environment. Due to the development of sensor technology, a more comprehensive information interaction function of the smart home has been realized, the life style has been optimized, and the safety of home life has been enhanced [18]. The principles of designing a smart home system are shown in Figure 1.

1. Convenience. The development of science and technology should be people-oriented, and the main purpose of the development of smart home is to make people live in a more comfortable, safe, and convenient environment [19]. Therefore, when designing a smart home system, the user's usage habits, especially the middle-aged and elderly groups, should be considered as much as possible, and a set of home control systems that are easy to operate should be designed.
2. Stability. In a productized smart home, it is not only necessary to ensure the stability of the system but also to ensure the stability of network transmission, hardware, and operation [20]. When designing a smart home system, it is necessary to fully consider the possible problems of each subsystem in the system. On the premise of ensuring the safety and stability of the system, solutions to the corresponding problems should also be given.
3. Interoperability. To ensure the compatibility between different products, the design of the smart home system needs to adopt a unified standard implementation. In terms of system communication, TCP/IP can be used as the communication protocol to ensure the compatibility between different products so that different products can be compatible and interconnected.
4. High-cost performance. Nowadays, housing prices are increasing year by year, and the cost of people's home environment is gradually increasing. If the cost of smart home systems is too high, it will not be easy for the public to accept. Therefore, it is very important to design a smart home system that meets system performance and low cost.
5. Intelligent. The designed smart home system should meet ergonomic needs, integrate self-learning technology, and pay more attention to people's living habits so that technology can serve people.

The article "The Design of the Lightweight Smart Home System and Interaction Experience of Products for Middle-Aged and Elderly Users in Smart Cities" was published in 2022. Journal: Comput Intell Neurosci.

### 3.2. Design of Smart Home System

A smart home system is designed, which is divided into two parts, namely hardware system and software system. The software system includes three parts: intelligent control subsystem, intelligent monitoring subsystem, and intelligent protection subsystem. The overall structure of the smart home system is shown in Figure 2. The intelligent control system is used to realize the intelligent control function, the intelligent monitoring subsystem is used to realize the intelligent security function, and the intelligent monitoring subsystem is used to realize the function of intelligent monitoring.

The intelligent control system is shown in Figure 3. There is a Kinect device in this module, through which the depth image information and human skeleton node information are collected. The position of the skeleton nodes is analyzed to obtain the human posture information so that the smart home equipment can be controlled. In the action recognition module, the function of dynamic gesture recognition is also added, which can be used to control the opening and closing of curtains and other devices by waving the arm in front of the Kinect device.

The structure of the intelligent monitoring subsystem is shown in Figure 4. The system is used to realize the intelligent security function. This module has a very excellent performance in recognizing small-scale actions, such as detecting someone falling or coughing violently at home, someone knocking on the door, climbing, and other behaviors. When the above abnormal behavior is detected, the module can send alarm information to the homeowner in time to avoid adverse consequences. The emphasis is on the introduction of the intelligent monitoring subsystem.

The structure of the intelligent security subsystem is shown in Figure 5. The system is used to realize the function of intelligent monitoring. As the material in today's society becomes more and more abundant, family sports and fitness have become a trend. The intelligent monitoring subsystem can well recognize the human–object interaction, and fitness generally requires fitness equipment, so it can supervise and correct the movement of family members. In addition, if someone at home needs to do rehabilitation training, this module can also be used to monitor whether the action is correct, thereby reducing labor costs.

The article "The Design of the Lightweight Smart Home System and Interaction Experience of Products for Middle-Aged and Elderly Users in Smart Cities" was published in 2022. Journal: Comput Intell Neurosci.

### 3.3. Intelligent Security Subsystem Based on the Small-Scale Motion Detection Algorithm

In general, small-scale motion has a small range of motion and may remain in a stationary state for a long time, so it is difficult to complete the detection. In past studies, researchers have mainly used handcrafted features to extract information from videos, such as directional optical flow histogram, directional gradient histogram, motion boundary histogram, and other descriptors to represent video information, which is used for express handcrafted features [21]. Handcrafted human behavioral features refer to people manually designing an image-encoding scheme based on human behavioral features observed in behavioral videos and image statistical features.

To improve the recognition of the original optical flow image, the more diverse human action information in the video is mined, and the information of the attention-enhanced image and the optical flow image is combined so that the detection performance of small-scale motion can be improved. In this regard, a new action recognition system is proposed. The specific process is shown in Figure 6. The system uses three 3D CNN to extract three image features so that the data information in the video can be fully extracted. The first step of the system is to use the Structural Similarity (SSIM) method to exclude images with high similarity in the dataset, calculate the optical flow images of the remaining images, and then enhance the features of the optical flow images [22]. Using the target detection method of Class Activation Map (CAM) that is used to obtain CAM-Mask, and then it is multiplied with Red Green Blue (RGB) image and optical flow image to obtain CAM-optical flow image and CAM-RGB image. Finally, the mixed image is obtained by Poisson fusion of the CAM-optical flow image and the original RGB image. The system uses three 3D ResNet-18 models to extract eigenvalues from CAM-optical flow images, CAM-RGB images, and mixed images. Then the three obtained feature matrices are added and fused into a feature matrix, and the fused matrix is sent to the classifier to complete the final classification. The designed classifier contains two fully connected layers and one support vector machine (SVM) layer.

The article "The Design of the Lightweight Smart Home System and Interaction Experience of Products for Middle-Aged and Elderly Users in Smart Cities" was published in 2022. Journal: Comput Intell Neurosci.

#### 3.3.1. Preprocessing of the Dataset

Preprocessing the dataset can improve the recognition of the optical flow image to a certain extent. The core of preprocessing is the SSIM algorithm, which is used to measure the similarity of images [23]. SSIM consists of luminance contrast *l*(*x*, *y*), contrast contrast *c*(*x*, *y*), and structural contrast *s*(*x*, *y*), and its equations are as follows:

(1) $$\begin{array}{c} ssim\left(x,y\right)={\left[l\left(x,y\right)\right]}^{\alpha }\times {\left[c\left(x,y\right)\right]}^{\beta }\times {\left[s\left(x,y\right)\right]}^{\gamma }, \end{array}$$

(2) $$\begin{array}{c} l\left(x,y\right)=\frac{2\mu_{x}\mu_{y}+C_{1}}{\mu_{x}^{2}+\mu_{y}^{2}+C_{1}}, \end{array}$$

(3) $$\begin{array}{c} c\left(x,y\right)=\frac{2\sigma_{x}\sigma_{y}+C_{2}}{\sigma_{x}^{2}+\sigma_{y}^{2}+C_{2}}, \end{array}$$

(4) $$\begin{array}{c} s\left(x,y\right)=\frac{\sigma_{xy}+C_{3}}{\sigma_{x}\sigma_{y}+C_{3}}, \end{array}$$

*x* and *y,* respectively, represent the pixel matrix of the two input images; (*μ*_*x*_, *μ*_*y*_) means the local mean of *x* and *y*; (*σ*_*x*_, *σ*_*y*_) denotes the variance of *x* and *y*; *σ*_*xy*_ indicates the covariance of *x* and *y*; *C*1, *C*2, and *C*3 are parameters, and the meaning of existence is to avoid the denominator being equal to 0. The values of *C*1, *C*2, and *C*3 are set to 1 × 10^−5^.

#### 3.3.2. Feature Enhancement Algorithm

A feature enhancement method that can further improve the recognition of optical flow image is proposed as shown in equations (5) to (7):

(5) $$\begin{array}{c} A=\text{IMG}-M, \end{array}$$

(6) $$\begin{array}{c} B=\text{CLIP}\left(A÷\left(S+X\right)\times 0\cdot 1+0\cdot 5\right), \end{array}$$

(7) $$\begin{array}{c} C=B\times 255. \end{array}$$

IMG expresses the pixel value matrix of the input image; *M* represents the average value of IMG; *S* refers to the standard deviation of *A*; *X* is a random number, and 0 < *X* < 1. The CLIP function restricts the value of matrix *B* to the [0, 1] interval; *C* denotes the matrix after feature enhancement.

### 3.4. ResNet Models

Deep residual network (ResNet) refers to the Visual Geometry Group (VGG) 19 network, modified it on the basis, and added a residual unit through a short-circuit mechanism [24, 25]. The change is mainly reflected in the fact that ResNet directly uses the convolution of stride = 2 for downsampling and replaces the fully connected layer with the global average pool layer. An important design principle of ResNet is that when the size of the feature map is reduced by half, the number of feature maps is doubled, which maintains the complexity of the network layers. The CNN used in the backbone of the system is 3D ResNet-18, while the CNN used in the grade-cam++ method is 2D ResNet-50.

The article "The Design of the Lightweight Smart Home System and Interaction Experience of Products for Middle-Aged and Elderly Users in Smart Cities" was published in 2022. Journal: Comput Intell Neurosci.

### 3.5. Experimental Dataset and Parameter Settings

The main source of video data in the University of Central Florida (UCF101) is collected from YouTube after editing, and the collected video data is divided into 101 types, each type of action contains 25 groups, and action of each type contains 25 groups. There are 4–7 fragments in each group [26]. UCF101 has a total of 13,320 videos. The resolution of these videos is 320*∗*240. Each action is obtained after multiple shooting in different shooting environments. The shooting environment includes appearance changes, background changes, camera movement, lighting changes, etc. The 101 types of actions can be roughly divided into three categories: human–object interaction videos, human motion videos, and videos that do not contain complete personal information.

The HMDB51 dataset contains a total of 6,849 videos, demonstrating a total of 51 actions, each action contains at least 51 videos, and the resolution of these videos is 320*∗*240 [27]. The data in HMDB51 is mainly from YouTube, Google Video, and other websites. The 51 types of actions are divided into three categories: human–object interaction actions, human actions, and facial actions.

In this experiment, UCF101 and HMDB51 are divided into two parts, two-thirds of which are training sets, and the remaining one-third are test sets. After processing the video frames using the SSIM algorithm, all frames in the training set are taken as input, and the input frames are scaled to a short size of [224, 224]. This experiment uses NVIDIA GTX 1080 GPU to train and evaluate the model, set the batch size to 16 and the learning rate to 0.001. After training for 26 or 27 epochs, the model can be further optimized only by reducing the learning rate. Therefore, the training process requires a total of 80 epochs. When the experiment goes to 30 epochs and 60 epochs, the learning rate is reduced to 0.1 times of the original. This experiment uses the PyTorch framework to implement all experiments.

The 2D ResNet used is ResNet-50 officially released by Pytorch, which can recognize a variety of objects including people and has relatively high accuracy in mainstream datasets. The three 3D Resnet-18 used in the system are trained on the UCF101 original RGB image dataset, the UCF101 optical flow image dataset and the mixed image dataset in turn.

## 4. Results and Discussion

### 4.1. Accuracy of Each Group within UCF101

UCF101 is divided into three groups, in which the action category of Group1 is human motion, the video of Group2 does not contain complete human information, and the action category of Group3 is human–object interaction. The average accuracy of each group is shown in Figure 7.

The article "The Design of the Lightweight Smart Home System and Interaction Experience of Products for Middle-Aged and Elderly Users in Smart Cities" was published in 2022. Journal: Comput Intell Neurosci.

In Figure 7, for the UCF101 dataset, the accuracy of the system in recognizing actions in Group1 is 94.64%, the accuracy of the system in recognizing actions in Group2 is 77.12%, and the accuracy in recognizing actions in Group3 is 41.51%. It indicates that the system has the best performance when recognizing actions within Group1.

### 4.2. Accuracy of Each Group within HMDB51

The HMDB51 is also divided into three groups, in which the action category of Group1 is human motion, the action category of Group2 is the interaction between people and objects, and the action category of Group3 is facial action. The average accuracy of each group is shown in Figure 8.

In Figure 8, for the HMDB51 dataset, the accuracy of the system in recognizing actions in Group1 is 90.11%, the accuracy in recognizing actions in Group2 is 29.51%, and the accuracy in recognizing actions in Group3 is 84.06%. It demonstrates that the system has the best performance in recognizing actions in Group1. The main reason is that the CAM-based target detection method can accurately detect human targets when detecting such actions. It enables the system to extract all the useful motion information in the action category and also removes the influence of background that the system can extract the action category.

### 4.3. Comparative Analysis of the Accuracy of Different Methods

The performance of the intelligent security subsystem based on the small-scale motion detection algorithm some of the most advanced action recognition methods are compared in the HMDB51 data set and the UCF101 data set, and action types such as eat, chew, wave have a high degree of similarity, short duration, and small range of motion, so they are difficult to identify. The comparison results of the designed intelligent security subsystem based on the small-scale action detection algorithm and other advanced methods in the small-scale action category are shown in Figure 9.

Figure 9 indicates that the recognition accuracy of the intelligent security subsystem based on the small-scale motion detection algorithm in the recognition of Hair-cut, Chew, Wave, Drink, Jump rope, and Hair-cut is 69.1, 52, 77.5, 72.3, 77.4, and 88.9%, respectively, which are much more accurate than other methods. The main reason is that other methods only use one or two pieces of information as the basis for action recognition, which cannot provide enough time–space dimension information, so they are limited in recognizing these actions. The designed intelligent security subsystem based on the small-scale action detection algorithm fully exploits time dimension information, space dimension information, and mixed spatiotemporal dimension information as the basis of action recognition, thus greatly improving the recognition accuracy of these action categories.

The article "The Design of the Lightweight Smart Home System and Interaction Experience of Products for Middle-Aged and Elderly Users in Smart Cities" was published in 2022. Journal: Comput Intell Neurosci.

The accuracy of the intelligent security subsystem based on the small-scale motion detection algorithm and other advanced methods in recognizing camera movement is compared and the results are shown in Figure 10.

Figure 10 refers that the proposed intelligent security subsystem based on the small-scale action detection algorithm has a recognition accuracy of 96.4, 92.3, and 85.4% in identifying the action categories of Diving, Skiing, and Swing, respectively. It means that the proposed intelligent security subsystem based on the small-scale motion detection algorithm can eliminate the influence of the background. In the case of camera movement, the recognition accuracy of the proposed intelligent security subsystem based on the small-range motion detection algorithm can be comparable to other advanced algorithms.

## 5. Conclusion

In recent years, action recognition technology based on computer vision has played an increasingly significant role in the fields of healthcare, HCI, and automated video surveillance. Therefore, the monitoring and HCI functions of image recognition in the smart home are deeply explored. A smart home system for middle-aged and elderly users is designed. To increase the security of the smart home, the intelligent monitoring subsystem is improved, and an intelligent security subsystem based on a small-scale motion detection algorithm is proposed. The proposed intelligent security subsystem based on a small-scale motion detection algorithm can maximize the temporal and spatial features in the video, improve the performance of the algorithm, and realize the intelligent security function based on human motion. The research results demonstrate that for the UCF101 dataset, the system has an accuracy of 94.64% in recognizing actions in Group1; for the HMDB51 dataset, the system has an accuracy of 90.11% in recognizing actions in Group1. The recognition accuracy of the intelligent security subsystem based on the small-scale motion detection algorithm in the recognition of Hair-cut, Chew, Wave, Drink, Jump rope, and Hair-cut is 69.1, 52, 77.5, 72.3, 77.4, and 88.9%, which are much more accurate than other methods. The recognition accuracy of the system in identifying the action categories of Diving, Skiing, and Swing is 96.4, 92.3, and 85.4%, respectively. In a word, the recognition accuracy of the proposed intelligent security subsystem based on the small-scale motion detection algorithm can be comparable to other advanced algorithms. The motion recognition technology is used in smart home systems to increase the safety and comfort of smart home by using computer vision technology. The disadvantage is that the existing target detection algorithms often consume a lot of computing resources, and target detection and feature enhancement cannot be performed at the same time, which slows down the running speed of the overall algorithm. Therefore, in future research, an algorithm that can simultaneously perform target detection and improve target area information will be designed.

The article "The Design of the Lightweight Smart Home System and Interaction Experience of Products for Middle-Aged and Elderly Users in Smart Cities" was published in 2022. Journal: Comput Intell Neurosci.

## Figures and Tables

**Figure 1:** Design principles of smart home systems.

**Figure 2:** The overall structure of the smart home system.

**Figure 3:** The structure of the intelligent control system.

**Figure 4:** The structure of the intelligent security subsystem.

**Figure 5:** The structure of the intelligent monitoring subsystem.

**Figure 6:** The process of action recognition subsystems.

**Figure 7:** Accuracy of each group within UCF101.

**Figure 8:** Accuracy of each group within HMDB51.

**Figure 9:** Accuracy comparison of small-scale action.

**Figure 10:** Accuracy comparison of camera movement actions.

## Data Availability

All data are fully available without restriction.
